# Development of a Novel Deep Learning-Based Prediction Model for the Prognosis of Operable Cervical Cancer

**DOI:** 10.1155/2022/4364663

**Published:** 2022-11-26

**Authors:** Taotao Dong, Linlin Wang, Ruowen Li, Qingqing Liu, Yiyue Xu, Yuan Wei, Xinlin Jiao, Xiaofeng Li, Yida Zhang, Youzhong Zhang, Kun Song, Xingsheng Yang, Baoxia Cui

**Affiliations:** ^1^Department of Obstetrics and Gynecology, Qilu Hospital of Shandong University, Jinan 250012, China; ^2^Department of Radiation Oncology, Shandong First Medical University and Shandong Academy of Medical Sciences, Jinan 250117, China; ^3^Cheeloo College of Medicine, Shandong University, Jinan 250012, China; ^4^Shandong University of Traditional Chinese Medicine, Jinan 250335, China

## Abstract

**Background:**

Cervical cancer ranks as the 4th most common female cancer worldwide. Early stage cervical cancer patients can be treated with operation, but clinical staging system is not a good predictor of patients' survival. We aimed to develop a novel prognostic model to predict the prognosis for operable cervical cancer patients with better accuracy than clinical staging system.

**Methods:**

A total of 13,952 operable cervical cancer patients were retrospectively enrolled in this study. The whole dataset was randomly split into a training set (*n* = 9,068, 65%), validation set (*n* = 2,442, 17.5%), and testing set (*n* = 2,442, 17.5%). Cox proportional hazard (CPH) model and random survival forest (RSF) model were used as baseline models for the prediction of overall survival (OS). Then, a deep survival learning model (DSLM) was developed for OS prediction. Finally, a novel prognostic model was explored based on this DSLM.

**Results:**

The C-indexes for the CPH and RSF model were 0.731 and 0.753, respectively. DSLM, which had four layers that had 50 neurons in each layer, achieved a C-index of 0.782 in the validation set and a C-index of 0.758 in the testing set. The novel prognostic model based on DSLM showed better performances than the conventional clinical staging system (area under receiver operating curves were 0.826 and 0.689, respectively). Personalized survival curves for individual patient using this novel model also showed notably different survival slopes.

**Conclusions:**

Our study developed a novel, practical, personalized prognostic model for operable cervical cancer patients. This novel prognostic model may have the potential to provide a more prognostic information to oncologists.

## 1. Background

In 2020, an estimated 604,127 new cases of cervical cancer were diagnosed and 341,831 deaths occurred worldwide due to this malignancy [1]. Cervical cancer was the 5th most common female malignancy (11.3%) and the 4th most common cause of cancer mortality (5.2%) in high/very high HDI countries; however, in low/medium HDI countries, cervical cancer was the 2nd most common type of cancer (13.8%) and the 2nd most common cause of cancer death (12.4%) among women [2]. Due to the development of cytology screening, more and more cervical cancer patients will be diagnosed as early stage. Standard treatment for early stage (IA-IIB) cervical cancer patients has been radical hysterectomy and/or bilateral pelvic lymphadenectomy. However, nearly 23% of operable cervical cancer patients will still die from this disease within 5 years after primary diagnoses [3]. Thus, improving patient survival is still the ultimate goal for the treatment of operable cervical cancer. Precise survival prediction could play an important role in clinical practice as it could identify those patients who could benefit more from aggressive treatment due to their worse survival probabilities [4]. In addition, precise survival prediction may help improve the quality of future clinical trials as it could reduce potential biases during the assignment of different treatments. However, an increasing number of studies have pointed out that the currently used FIGO (Federation International of Gynecology and Obstetrics) clinical staging system for cervical cancer could not provide very accurate prognostic information for cervical cancer patients [5–7]. Thus, a novel prognostic model for operable cervical cancer is urgently needed.

The Surveillance, Epidemiology, and End Results (SEER) database covers nearly 28% of the total U.S. population and is the only population-based comprehensive cancer dataset [8]. SEER registers have been collecting demographic and clinicopathological data of cancer patients since 1973. Various studies have used the SEER dataset to perform survival analyses for different types of cancers, including cervical cancer [9–11]. However, nearly all of these studies used the Cox proportional hazard (CPH) model for analyses. Such studies have not effectively handled nonlinear correlations between risk factors and survival outcomes that are more common in the real world.

Deep learning methods can identify nonintuitive and complex relationships in data and are especially powerful for large datasets [12]. Deep learning methods have been explored in various medical settings, including radiologic image readings: characterization broadly captures the segmentation, diagnosis, and staging of tumors [13]; pathological diagnoses: a multiple instance learning-based deep learning system on whole slide images to diagnosis prostate cancer, basal cell carcinoma, and breast cancer metastases to axillary lymph nodes [14]; and treatment response predictions: a Deep Neural Network (DNN) was created to predict complete response after neoadjuvant rectal chemoradiotherapy, with an 80% accuracy [15]. However, studies involving the application of deep learning to cancer prognostication are rather limited.

In this study, we explored the potential of the deep learning method in predicting the survival rates of operable cervical cancer patients enrolled from the SEER dataset. In addition, we tried to develop a novel prognostic model based on the established deep learning model for operable cervical cancer, and personalized survival curves for patients from this novel prognostic model were also plotted.

## 2. Methods

### 2.1. Data Collection

The SEER database is a longitudinal dataset that collected data from 17 population-based cancer registers. Data from these registers will be desensitized every two years. Then, data will be submitted to the National Cancer Institute and will be utilized by researchers worldwide. The original dataset has 133 usable variables [8].

In this study, we used the “International Classification of Disease for Oncology, Third Edition (ICD-O-3)” for the selection of primary cervical cancer patients diagnosed from 1973 to 2014. The selection codes for ICD-O-3 were C53.0 (endocervix), C53.1 (exocervix), C53.8 (overlapping lesion of cervix uteri), and C53.9 (cervix uteri). Inclusion criteria include the following: patients were diagnosed with stage IA to stage IIB cervical cancer confirmed by histopathology according to the FIGO staging system 2019. Exclusion criteria are patients with (1) patients who had multiple tumors; (2) patients not having surgery; (3) patients not having follow-up data.

The more variables we input into our deep learning model, the more robustness the model becomes. Compared with nonoperable cervical cancer patients, operable cervical cancer patients have more clinicopathological variables, such as the depth of invasion, the number of dissected lymph nodes, the number of positive lymph nodes, and surgery type. Our main purpose is to prove deep learning model is superior to conventional staging system, so we selected operable cervical cancer patients, as they have more clinicopathological variables. Thus, patients with stage IA-IIB disease were selected for this study. Stage selection was based on “SEER Extent of Disease, 1988: Codes and Coding Instructions.” The final sample size was 13,952.

Because patients cannot be identified, the research ethics board of the Qilu Hospital of Shandong University exempted this study from review. However, a data use agreement submission was required to access the SEER Research Data File. We submitted the data agreement form to the SEER administration. Upon acceptance of the agreement, the SEER^∗^Stat software and data files were downloaded directly from the SEER website.

### 2.2. Preparation of Research Data

Based on our prior medical knowledge, the selected variables for further analyses were age, depth of invasion, year when patients were diagnosed, diameter, differentiation, histology, lymph node metastases, number of positive lymph nodes, number of dissected lymph nodes, marital status, primary tumor site, race, stage, and surgery type. We excluded those duplicated variables using correlation matrix analyses, and setting correlation coefficient threshold: 0.7.

Stages, lymph node metastases (no metastases, pelvic lymph node metastases, or para-aortic lymph node metastases), depth of invasion (depth less than 1/3, depth between 1/3 and 2/3, and depth deeper than 2/3), and histology (squamous, adenocarcinoma, or other types) were defined as categorical variables. The number of positive lymph nodes and the number of dissected lymph nodes were defined as continuous variables. Diameters were also defined as continuous variables. The differentiation variable has three types: poor, moderate, or well differentiation.

### 2.3. Deep Survival Neural Network

The deep survival neural network in this study was developed based on a neural multitask logistic regression (N-MTLR) model. The N-MTLR model was first developed by Fotso in the paper “Deep neural networks for survival analysis based on multitask framework” [16]. The original multitask logistic regression model was first introduced by Yu et al. in the paper “Learning patient-specific cancer survival distributions as a sequence of dependent regressors” [17]. The community code can be found in https://paperswithcode.com/paper/deep-neural-networks-for-survival-analysis.

Overall survival was defined as patient outcomes, which were measured by interval time between diagnoses and death, as well as the occurrence of event (death will be annotated as 1, while alive will be annotated as 0). If another patient had been lost during follow-up, then this patient will be annotated as censored, we will exclude this patient in next analysis process.

First, DSLM was applied to the stage IA-IIB cervical cancer dataset to make the prediction. Thereafter, patient samples were classified into five subgroups with different prognostic statuses, namely newtype1-5, according to the values of the risk scores.

### 2.4. Evaluation of Models and Statistical Analyses

We used the Concordance index (C-index) to measure the performances of different models. The C-index represents the global assessment of the model discrimination power; this is the model's ability to reliably provide a ranking of the survival times based on the individual risk scores. In general, when the C-index is close to 1, the model has an almost perfect discriminatory power; but if it is close to 0.5, it has no ability to discriminate between low- and high-risk patients. The *P* values were calculated through a *z*-score test proposed by Kang et al. [18], the difference was considered significant if the *P* value was less than 0.05. We also used the Brier scores to evaluate model performances. The Brier scores measure the average discrepancies between the true and the estimated probabilities at a given time. The lower the score (usually below 0.25), the better the model performance. To assess the overall error values across multiple time points, the integrated Brier scores (IBS) will be computed as well. Finally, median absolute error and mean absolute error measure the difference between the predicted and reality number of events (death) in each time window was also measured.

In the testing set, Kaplan-Meier curves for patients staged with the conventional staging model were drawn. Additionally, Kaplan-Meier curves using the novel prognostic model were plotted. Log-rank tests were used for the comparison of different curves, the difference was considered significant if the *P* value was less than 0.05. Receiver operating characteristics (ROC) and area under curves (AUC) were used for the comparison of prediction accuracy of conventional and novel prognostic model. The *P* values were calculated through *z*-score test, the difference was considered significant if the *P* value was less than 0.05. The deep learning model was developed on the Pytorch framework. Scikit-learn and pandas packages were also used for the treatment of data. We also used Stata software (StataCorp, 2015, Stata: Release 14. Statistical Software, College Station, TX, USA) and R software (version 3.0, R Foundation for Statistical Computing, Vienna, Austria) for other statistical analyses.

## 3. Results

### 3.1. Patient Demographics and Characteristics

A total of 13,952 cases of primary operable cervical cancer registered from 1973 to 2014 were enrolled in this study (Figure 1). The correlation matrix was plotted for 15 selected variables. The correlation coefficient between these variables, which we select all less than 0.7 (Figure 2), show that none of the variables we selected were duplicated.

The whole SEER dataset was split into a training set (*n* = 9,068, 65%), validation set (*n* = 2,442, 17.5%), and testing set (*n* = 2,442, 17.5%). The patient demographic characteristics are shown in Table 1. A total of 10,927 cases were white, 1,417 were black, and 1,379 were Chinese. A total of 5,967 cases were staged as IA (42.8%), 5,999 cases were IB (43.0%), 662 cases were IIA (4.7%), and 1,243 cases were IIB (8.9%). A total of 9,971 cases had squamous cell type (71.5%), 2,501 cases were adenocarcinoma types (17.9%), and 1,480 cases were other types (10.6%). Poor, moderate, and well differentiation tumors accounted for 24.9%, 25.1%, and 10.2%, respectively. A total of 3,208 cases (23%) died from all possible causes during the follow-up period. The overall 5-year survival for this cohort of patients was 84.5%.

### 3.2. Baseline Survival Prediction Models

The CPH model was first developed for comparison. In this study, a C-index of 0.731 was achieved in a 5-year survival prediction using the CPH model. In addition, the CPH model in this study had an IBS of 0.12 (Figure 3(a)).

We then developed another common machine-learning model: the random survival forest (RSF) model. Random survival forests are an ensemble learning method for classification that operate by constructing a multitude of decision trees at training time and outputting the class that is the mode of the classes output by individual trees. RSF achieved a C-index value of 0.753. Additionally, IBS was 0.13 for RSF (Figure 3(b)). All potential risk factors were ranked by their importance as follows Table 2: stage, lymph node metastasis, diameters, marital status, age, depth of invasion, surgery types, number of positive lymph nodes, differentiation, race, year when patients were diagnosed, histology, number of resected lymph nodes, Hispanic ethnicity, and primary tumor sites.

### 3.3. Training and Validation of a Deep Survival Learning Model (DSLM)

Patient survival belongs to time-to-event data, which cannot be handled by the classic deep learning method. Here, we used a “multitask logistic regression model” for tackling the censored data, which could represent patient-specific survival data as a sequence of dependent regressors (https://arxiv.org/pdf/1801.05512).

The final established deep learning network had four layers, in which layer 50 neurons were used (Figure 4). The ReLU activation method was used for each layer. The grid searching method was used for the selection of optimal hyperparameters. In addition, the l2 regularization and dropout method were used to prevent overfitting. The selected optimal hyperparameters were as follows: initial method was Glorot uniform, optimizer was Adam, learning rate was 1e-4, l2 regularization was 1e-2, l2 smooth was 1e-2, and dropout rate was 0.2. The values of the loss function decreased from 20,000 to 11,794 after 2000 iterations (Figure 5(a)). Finally, our model reached 0.782 for the C-index and 0.11 for IBS in the validation set (Figure 5(b)).

In this study, our DSLM achieved a median absolute error of 7.712 and a mean absolute error of 8.612 during sequential time intervals in the validation set (Figure 5(c)). Thus, all of these metrics suggested that DSLM could achieve acceptable discriminative power in survival prediction.

### 3.4. Further Evaluation of DSLM in the Testing Set

To prevent potential overfitting of DSLM, we also evaluated the performance of DSLM using a testing set. DSLM could resist this testing with a C-index of 0.758 (DSLM vs. CPH, *P* < 0.01; DSLM vs. RSF, *P* < 0.01) and IBS of 0.12 (Figure 6(a)). Additionally, DSLM provided good overall results over the entire 275 months of follow-up in the testing set. It only made a median absolute error of ~7 patients (Figure 6(b)).

In addition, calibration survival curves were also drawn using DSLM in this testing set. Calibration curves showed that nearly all parts of the predicted survival curves were plotted within regions between the lower and upper confidence ranges of the actual survival curves (Figure 6(c)). In other words, we could confidently draw the conclusion that predicted survival curves could represent actual survival probabilities in this study.

### 3.5. Novel Cervical Cancer Prognostic Model Based on DSLM

Risk factors for each patient in the testing set were then computed by our DSLM. Then, patients were divided into five prognostic groups according to their risk scores (Figure 7). The performances of commonly used clinical staging models and these novel prognostic methods were then compared.

Kaplan-Meier curves were plotted for patients from conventional staging stages, i.e., stage IA, IB, IIA, and IIB (Figure 8(a)). In addition, the difference in survival of these patients was significant (log rank test, *P* < 0.05). In addition, mortality for patients staged IB, IIA, and IIB increased 2.2-, 6.4-, and 7.5-fold relative to patients staged IA in Cox regression analysis.

Survival curves of patients stratified using the novel prognostic model were also plotted (Figure 8(c)), in which the difference in survival probabilities had achieved significance (*P* < 0.05). Additionally, mortality for patients with novel prognostic type 2, 3, 4, and 5 disease increased 4.6-, 20.9-, 46.9-, and 92.3-fold relative to patients with novel prognostic type 1 disease, respectively. Please note that survival outcomes of patients using novel type 1 are much better than those from commonly used clinical stage 1A, while survival for patients from novel type 5 are worse than those from clinical stage IIB.

For the concordance index, the performances of the novel prognostic model were also superior to those of the clinical staging model (novel prognostic vs. clinical staging: 0.782 vs. 0.682, *P* < 0.01). Receiver operating characteristic (ROC) curves for detecting death cases were also plotted for these two models. The area under the curve (AUC) of the ROC curve was 0.689 for the clinical staging model (Figure 8(b)), while the AUC of the novel prognostic model was 0.826, *P* < 0.01 (Figure 8(d)).

### 3.6. Personalized Survival Prediction Using DSLM

Our DSLM is very suitable for personalized survival prediction since it inherently could represent follow-up time as a series of time points.  Figure 9 shows five survival curves for five patients randomly selected from the testing set using our novel prognostic model. The slopes of these five curves were notably different, which reflected the difference in death risks between these patients, patients with low-risk had the best survival result, contrasting with patients with high-risk resulting in short survival time. This personalized usage of DSLM suggested that our model may have potential implications in this personalized cancer treatment era.

## 4. Discussion

To the best of our knowledge, this is the first cervical cancer prognostication study that takes advantage of a population-based dataset and a cutting-edge deep learning method. Various studies have explored the potential of deep learning in cervical cancer research, which includes cytology tests [19, 20], radiologic diagnoses [21, 22], and genetic data analyses [23, 24]. However, the potential of deep learning methods in cervical cancer survival prediction is largely unknown. Our DSLM showed a better C-index of 0.782 and IBS of 0.11 when compared to the conventional CPH or RSF model in the analyses of survival data.

In addition, the performance of our novel prognostic model is superior to that of the commonly used clinical staging model (ROC of death rate detection for the novel prognostic model vs. that of the clinical staging model: 0.826 vs. 0.689). Two possible reasons could account for this better performance: (1) more demographic and pathological factors have been included in this novel prognostic model. Indeed, Zeng et al. found that the performance of the cervical staging model could be improved by incorporating more pathological factors [25]. (2) We also show for the first time that the deep learning method could play an important role in the prognostication of cervical cancer patients.

In addition, our DSLM could provide personalized survival prediction for cervical cancer patients. Zhang et al. utilized age, race, pathological types, histology grades, radiotherapy, and chemotherapy to construct a nomogram for cervical cancer survival prediction [5]. Additionally, our group once developed nomograms for esophageal and lung cancer prognostication [26, 27]. However, these nomograms have two limiting drawbacks. First, the development of a nomogram is mainly based on logistic or CPH assumptions, which cannot capture nonlinear correlations between risk factors and survival outcomes. Second, the number of risk factors included in the nomogram is rather limited. Thus, the performances of such nomograms are readily easy to saturate. Therefore, it is believed that models such as DSLM could replace nomograms in near future cancer prognostication.

Superiority of this DSLM-based prognostic model is summarized as follows. This DSLM can directly learn patient characteristics from raw datasets without any kind of feature selection or engineering. In other words, such a model could incorporate different types of data comprehensively, including clinical, hematological, pathological, and genetic information. In addition, our DSLM is in fact a kind of dynamic model that could be further improved with the advent of novel incoming data or data from other large cancer centers.

There are several limitations in this study. First, the SEER dataset only has a limited number of clinicopathological factors. Second, visualization of the developed DSLM was not performed in this study due to the limited number of included variables. Thus, this DSLM is a kind of “black box” model, which may cause some confusion to clinicians when it will be utilized in clinical practice. Indeed, Matsuo et al. once identified several novel risk factors for cervical cancer patients through visualization of a developed model, which had not been recognized by conventional CPH [28]. Third, external validation of DSLM is urgently needed. It is unclear whether DSLM is suitable for patients from other regions or other ethnicities because all enrolled patients were mainly from the U.S. population and SEER database.

In summary, DSLM is a novel population-based deep survival learning model for cervical cancer patients. A novel prognostic model based on DSLM is proposed in this study, which has much better performance than the clinically used cervical cancer-staging model. It is believed that the deep learning method, multimodal integration, and big data are three cornerstones in future precision cervical cancer treatment.

## 5. Conclusions

This is the first study, which took advantage of Surveillance, Epidemiology, and End Results (SEER) dataset as well as deep learning method to develop a novel-staging model for operable cervical cancer patients. 13,952 cases of operable cervical cancer patients staged from IA to IIB were retrospectively enrolled in this study. A novel-staging model based on deep learning method showed better performances than conventional clinical staging model in mortality prediction, which had area under receiver operating curves (ROC) of 0.826 and 0.689, respectively. Last, personalized survival curves for patients from each novel stage could also easily plotted using this deep learning method.

## Figures and Tables

**Figure 1:** A workflow of data download and preprocessing.

**Figure 2:** Correlation matrix of 15 selected features. Values in this matrix indicate the correlation coefficient of two corresponding variables. Color indicates strength of correlation, in which dark blue and dark red indicate strong positive and strong negative relationships, respectively. Diag: the year when the patient was diagnosed; Diff: differentiation; Hist: histology; Lymmeta: lymph node metastasis; Lymno: numbers of resected lymph nodes; Lympo: number of positive lymph nodes; Primasite: primary tumor sites.

**Figure 3:** Baseline survival prediction models. (a) The CPH model had a prediction error curve with IBS (*t* = 272.0) =0.12. (b) The RSF model had a prediction error curve with IBS (*t* = 275.0) =0.13.

**Figure 4:** A workflow of DSLM development.

**Figure 5:** Training and validation of DSLM.. (a) The values of the loss function for DSLM decrease from 20,000 to 11,794 after 2000 iterations. (b**)** The prediction error curve with IBS (*t* = 272.8) =0.11 for DSLM. (c) Sequential values of actual and predicted number of patient deaths for each time interval in validation set. The red line indicates the actual number of patient deaths, while the blue line indicated the predicted number of patient deaths. The median absolute error equals to 7.712, while the mean absolute error equals to 8.612.

**Figure 6:** Further evaluation of DSLM in the testing set. (a) Prediction error curve with IBS (*t* = 272.8) =0.12. (b) Sequential values of actual and predicted number of patient deaths for each time interval in test set. The red line indicates the actual number of patient deaths, while the blue line indicated the predicted number of patient deaths. The median absolute error equals to 7.354, while the mean absolute error equals to 8.180. (c) The calibration curves of the actual and predicted number of remaining patients for each time interval in test set. The red line indicates the actual number of patient deaths, while the blue line indicated the predicted number of patient deaths. The median absolute error equals to 18.242, while the mean absolute error equals to 20.701.

**Figure 7:** Novel cervical cancer prognostic model based on DSLM. Five groups of patients based on risk scores estimated by DSLM. Thus, each patient is assigned a novel prognostic value. The left panel indicates the overall risk score distribution of enrolled cervical cancer patients. The right panel indicates the five groups of patients based on their risk scores stratified with DSLM.

**Figure 8:** Prognostic performance of DSLM is superior to conventional staging model. (a) Kaplan-Meier curves of patients staged with the clinical staging model. (b) ROC curves for the prediction of death rates using the clinical staging model. (c) Kaplan-Meier curves of patients stratified using the novel prognostic model based on our DSLM. (d) ROC curve for the prediction of death rates using the novel prognostic model based on our DSLM.

**Figure 9:** Personalized survival prediction using DSLM. Personalized patient survival curve for five patients selected from our novel prognostic model. In this figure, 5 patients in different risk groups were selected (in different colors), who clearly have different prognosis demonstrated in these survival curves.

**Table 1:** Patient demographic and clinicopathological characteristics.

Features	Characteristics	No.	%
Age (years)	Mean	43.0	
	SD	13.0	

Race	White	10927	78.3
	Black	1417	10.2
	American Indian	108	0.8
	Chinese	1379	9.9
	NA	121	0.8

Marital status	Single	3204	23.0
	Married	7340	52.6
	Separated	241	1.7
	Divorced	1636	11.7
	Widowed	901	6.5
	NA	630	4.5

Primary site	Endocervix	2520	18.0
	Exocervix	10978	78.7
	Overlapping lesion	454	3.3

Stage	IA	5967	42.8
	IB	5999	43.0
	IIA	662	4.7
	IIB	1243	8.9
	NA	81	0.6

Lymph node metastasis	No metastasis	11175	80.1
	Regional lymph node	1264	9.1
	Aortic/distant lymph node	202	1.4
	NA	1311	9.4

Positive lymph node numbers	0	11427	81.9
	1	1130	8.1
	2	530	3.8
	3	183	2.4
	4	334	1.3
	> = 5	348	2.5

Resected lymph node numbers	Mean	10.8	
	SD	13.7	

Tumor diameter (mm)	Mean	23.8	
	SD	33.1	

Depth of invasion	Inner 1/3	4141	29.7
	Middle 1/3	1100	7.9
	Outer 1/3	2210	15.8
	NA	6501	46.6

Histology	Squamous	9971	71.5
	Adenocarcinoma	2501	17.9
	Other types	1480	10.6

Differentiation	Poor	3475	24.9
	Moderate	3505	25.1
	Well	1416	10.2
	NA	5556	39.8

Surgery	Local excision	2466	17.6
	TH	1632	11.7
	TH + LND	838	6.0
	TH + BSO + LND	1953	14.0
	RTH + BSO + LN	7073	50.7

NA indicates not available.

**Table 2:** Ranking of all potential risk factors by RSF.

Number	Features	Importance	Percentage importance
0	Stage	7.546688	0.103754
1	Lymph node (LN) metastasis	7.514835	0.103316
2	Diameter	7.334223	0.100833
3	Marital status	7.309901	0.100498
4	Age	6.781088	0.093228
5	Depth of invasion	6.568536	0.090306
6	Surgery types	6.245984	0.085871
7	No. of positive LN	4.895398	0.067303
8	Differentiation	4.602522	0.063277
9	Race	3.959236	0.054433
10	Diagnoses year	3.567483	0.049047
11	Histology	2.917354	0.040109
12	No. of dissected LN	1.848070	0.025408
13	Hispanic ethnicity	1.645153	0.022618
14	Primary sites	-0.275462	0.000000

## Data Availability

Surveillance, Epidemiology, and End Results (SEER) Program is a long-established resource that allows for population-based surveillance and analysis of all cancers in the United States. The datasets analyzed during the current study are available on the (https://www.seer.cancer.gov). The SEER^∗^Stat software and data files can download directly from the SEER website.

## Abbreviations

CPH: Cox proportional hazard
RSF: Random survival forest
OS: Overall survival
DSLM: Deep survival learning model
AUC: Area under curves
SEER: The surveillance, epidemiology, and end results
FIGO: Federation International of Gynecology and Obstetrics
ICD-O-3: International Classification of Disease for Oncology, Third Edition
IRB: Institutional Review Board
N-MTLR: Neural multitask logistic regression model
IBS: Integrated Brier scores
ROC: Receiver operating characteristics
HDI: Human Development Index.
